RETRACTED

# The microRNA-1246 promotes metastasis in non-small cell lung cancer by targeting cytoplasmic polyadenylation element-binding protein 4

**DOI:** 10.1186/s13000-015-0366-1

**Published:** 2015-07-25

**Authors:** Weihua Huang, Huifen Li, Rongcheng Luo

**Affiliations:** TCM-Integrated Hospital, Southern Medical University, Cancer Center, NO.13 Shiliugang Road, Haizhu District, Guangzhou, Guangdong 510315 China; Department of Chemotherapy, Zhongshan People’s Hospital, Zhongshan, Guangdong 528400 China

**Keywords:** miR-1246, CPEB4, NSCLC, Metastasis

## Abstract

**Background:**

The microRNAs present a class of non-coding RNAs which are usually implicated in tumor biology. Recent report has unraveled that a novel member of microRNA family called miR-1246. However, the functional role and molecular mechanisms of miR-1246 in non-small cell lung cancer (NSCLC) is still elusive.

**Methods:**

Using RT-PCR, luciferase reporter, mRNA microarrays, invasion and migration assays, we investigated the potential role of miR-1246 in the pathogenesis of NSCLC.

**Results:**

In this study, we showed that miR-1246 markedly promoted NSCLC cell migration and invasion. Meanwhile, we found that cytoplasmic polyadenylation element binding protein 4 (CPEB4) might be involved and serve as a direct target of miR-1246 in NSCLC. *CPEB4* knockdown substantially enhanced NSCLC migration and invasion resembling the effect of miR-1246 in NSCLC. CPEB4 is also frequently downregulated in NSCLC and decreased CPEB4 expression correlated with poor survival.

**Conclusions:**

These results suggested that the miR-1246 may promote cell metastasis by targeting *CPEB4*. Meanwhile, the level of *CPEB4* could be used as a potential marker in NSCLC patients. Our findings unraveled novel functions of miR-1246 in lung cancer cells and shed light on NSCLC prognosis.

**Electronic supplementary material:**

The online version of this article (doi:10.1186/s13000-015-0366-1) contains supplementary material, which is available to authorized users.

## Background

Lung cancer is the leading cause of cancer-related mortality worldwide [1]. Lung cancer has been traditionally subdivided into two principal groups, namely, neuroendocrine and non-small cell lung cancer (NSCLC). The latter type is more common than the former. Cancer occurs and develops as a complicated result of an accumulation of various endogenous and exogenous effects. Gene alterations participate in cancer genesis. Alterations in many onco3 genes and tumor suppressor genes have been reported in lung cancer.

MicroRNAs (miRNA) are small noncoding RNA molecules that primarily serve as a posttranscriptional factor for gene expression. The miRNA can also function by base-pairing with the 3’-untranslated region (3’-UTR) of specific mRNAs [2]. Aberrant expression of miRNAs are often regarded as biomarkers of biological pathways leading to the occurrence of malignancy including cancer [3]. Many recent reports have clarified critical roles for miRNAs in regulating tumor cell invasion, metastasis and migration [4]. It is well known that miRNAs can participate in numerous biological processes, such as apoptosis, differentiation and invasion. During tumorigenesis, miRNAs may act either as an oncogene or a tumor suppressor and contribute to tumor initiation and progression by regulating specifically matched target genes. The miRNA functions in tumorigenesis and metastasis by directly targeting oncogenes or tumor suppressor genes [5, 6]. Different miRNAs may either function as oncogenes or tumor suppressors [7–10].

RETRACTED

Current knowledge of miRNA expression patterns and function in normal or neoplastic cells is just starting. The miRNA genes are usually located at fragile sites, as well as in minimal regions of amplification or common breakpoint regions, suggesting that miRNAs might be a new class of genes involved in human tumorigenesis [11]. For example, miR-15-a and miR-16-1 are frequently deleted and deregulated in patients with B cell lymphocytic leukemia [12]. Other association between cancer and miRNAs have been studied, including reduced expression of miR-143 and miR-145 in colorectal cancers [13] and let-7 in lung cancers [14], high expression of the precursor miR-155 in Burkitt’s lymphomas [15], and oncogenic function of miR-17-92 cluster in human B cell lymphomas as well as in lung cancers [16–18]. Recently, miR-1246 has been identified through a microRNA array and is potentially important for tumorigenesis [19]. However, the exact role of miR-1246 in lung cancer is currently unknown.

In this study, we showed that the expression of miR-1246 is significantly upregulated in lung cancer tissues compared with noncancerous tissues. Ectopically expressed miR-1246 could promote the migration and invasion of lung cancer cells. Furthermore, we found that CPEB4 is a direct and functional target of miR-1246. The expression of CPEB4 is closely correlated with therapeutic outcomes in NSCLC patients.

## Methods

### Lung cancer samples and cell lines

NSCLC tumor samples and noncancerous adjacent tissues (NAT, at least 3 cm from the tumor) were obtained from the surgical specimen archives of the TCM-Integrated Hospital, Southern Medical University. Our study was approved by the Ethical Committee of TCM-Integrated Hospital, Southern Medical University, and every patient had written informed consent, the study methodologies conformed to the standards of the Declaration of Helsinki. All lung cancer cell lines were purchased from Shanghai Institutes for Biological Sciences, Chinese Academy of Sciences and cultured according to the instructions (A549, H460, H1299, H226, H522, H596 and SW-900). Transfection was carried out and evaluated as described previously [20].

RETRACTED

### RNA extraction and quantitative real-time PCR

RNA isolation from cells or tissue samples was performed with the mirVana miRNA Isolation Kit (Ambion, Austin, TX) according to the manufacturer’s protocol. For RT-PCR detection of miR-1246 oligonucleotide, mature miR-1246 was reverse- transcribed with specific RT primers. Reverse transcription was performed using poly (A)-tailed total RNA and reverse transcription primer with ImPro-II Reverse Transcriptase (Sigma, Shanghai) as described previously [21]. The raw data were normalized by U6 small nuclear RNA using TaqMan miRNA assays (Applied Biosystems, Shanghai).

### Vector constructs

The lentivirus vector for miR-1246 expression pWPXL-miR-1246, the primary miRNA sequence amplified from normal genomic DNA replaced the green fluorescent protein fragment of the pWPXL mock vector. In the luciferase reporter, the wild-type or mutant 3’UTR of *CPEB4* was cloned downstream of the stop codon in the luciferase. Other potential target genes were cloned in a similar manner. The sequences of the primary miRNA and wild-type and mutant 3’ UTR were confirmed by sequencing.

### Lentivirus production and transduction

Virus particles were harvested from HEK 293 T cells 48 h after pWPXL-miR-1246 transfection with the envelope plasmid pMDG2 and the packaging plasmid psPAX2 using Lipofectamine 2000. A549 and H226 cells were infected with recombinant lentivirus-transducing units and 6 μg/mL polybrene.

### Transfection of oligonucleotide

The miRNA mimics and small interfering RNAs (siRNA) targeting *CPEB4* were designed and synthesized by GenePharma (Shanghai, China). The miR-1246 inhibitor was synthesized by RiboBio (Shanghai, China). Cells were transfected with mimic or inhibitor using Lipofectamine 2000, while siRNA transfection was performed with Lipofectamine RNAi MAX reagents according to the manufacturer’s instructions (Invitrogen, Shanghai). The transfection efficiency of miR-1246 mimics and inhibitors were verified and the inhibition can reach around 90 % (Additional file 1: Figure S1, A and B). Usually, after 72 h’ transfection, the cells were collected and used in further experiments. The sequences for the siRNAs were shown as follows:

**Table:** 

Si-CPEB4-1:	Sense	5′-CUGCCUCAUUUGGCGAAUAC-3′
	Antisense	5′-UAUUCGCCAAAUGAGGCAGC-3′
Si-CPEB4-2:	Sense	5′-CCUGCUGUUUCAAGAUGAAC-3′
	Antisense	5′-UUCAUCUUGAAACAGCAGGC-3′
Si-CPEB4-3:	Sense	5′-GCAGCAUGGAGAGAUAGAUC-3′
	Antisense	5′-AUCUAUCUCUCCAUGCUGCC-3′

RETRACTED

### Proliferation assay

The proliferation of specific cells was assessed by the Cell Counting Kit-8 (CCK-8) assay kit (Invitrogen, Shanghai, China). Approximately 10^4^ cells were seeded in each well of a 96-well plate, and 10 μL CCK-8 was added to 90 μL culture medium. After incubation at 37 °C for 2.5 h, the absorbance was detected at 450 nm and the OD450 value is correlated with live cell numbers.

### Migration and invasion assays

The migration and invasion assays were performed using a 24-well transwell plate (8-μm pore size, Corning, New York, USA). 4 × 10^5^ cells suspended in serum-free DMEM were appended to the upper chamber lined with non-coated membrane. For invasion assay, chamber inserts were coated with 2 μg/ml of Matrigel. DMEM containing 20 % FBS were added to the lower chambers as a chemoattractant. After 48 h transfection, the non-filtered cells were removed from the system with a cotton swab. Filtered cells located on the lower side of the chamber were stained with 0.2 % crystal violet (Sigma, Shanghai) for 0.5 h and then counted with a microscope (Olympus Corp., Tokyo, Japan).

### Luciferase reporter assay

HEK 293 T cells (293 T) were cultured in 96-well plates and transfected with 50 ng pluc-3’ UTR, 10 ng Renilla and 5 pmol miR-1246 mimic or negative control. After 72 h of incubation, the luciferase activity was determined using a dual-luciferase reporter system (Promega, Shanghai).

### Immunoblot

Cell lysates were prepared with 10 % SDS-PAGE and then transferred to the nitrocellulose membrane. The membrane was incubated with a rabbit anti-CPEB4 polyclonal antibody (Sigma, Shanghai), mouse anti-β-actin (Sigma, Shanghai) or mouse anti-GAPDH monoclonal antibody (Sigma, Shanghai). The proteins were displayed with chemi-luminescence reagents (Thermo Scientific, Hudson, NH, USA).

### Immunohistochemical Staining (IHC)

Tumor tissues were fixed in formalin and embedded in paraffin using the Microm Tissue Embedding Center (Labequip, Ltd, Markham, Ontario). Then the secretions were cut (5 μm) and stained with H&E. For immunohistochemical staining, sections were hydrated and blocked with 4 % H_2_O_2_ in water for 15 min. Antigen retrieval was done with 20 μmol/L citrate buffer (pH 6.0) for 15 min followed by a 20-min cooldown and washed in TBS with Tween (TTBS: 50 μmol/L Tris–HCl (pH 7.5), 150 mmol/L NaCl, 0.1 % Tween 20). Slides were treated with Biocare blocking reagent (Biocare Medical) for 15 min to remove nonspecific binding. Slides were then incubated with antibodies against *CPEB4* (Sigma, Shanghai) for 40 min. Then the slides were washed in TTBS for 40 min at 20 °C. After washing, the slides were incubated with antigoat horseradish peroxidase-conjugated secondary antibodies (BioGenex, San Francisco) for 40 min at 20 °C.

RETRACTED

### Statistical analysis

Statistical analysis was carried out using SPSS 16.0 software (SPSS Inc.; Chicago, IL, USA). Survival curves were constructed with the Kaplan-Meier method and compared by log-rank tests. The two-tailed Student *t* test was used for the other data analyses. The *p* values less than 0.05 were considered significant. Asterisks were used to represent statistical significance of *p* values in some figures, e.g. * *p* < 0.05, ** *p* < 0.01, *** *p* < 0.001.

## Results

### The miR-1246 is frequently upregulated in NSCLC and accelerates NSCLC cell migration and invasion

To confirm the expression of miR-1246 in NSCLC, we detected mature miR-1246 in 50 pairs of NSCLC and matched noncancerous adjacent tissues by real-time PCR. The results indicated that miR-1246 expression was upregulated in NSCLC tissues compared with the noncancerous tissues (Fig. 1a). A miR-1246 mimic was transfected into two NSCLC cell lines to determine whether it could affect cell proliferation and motility. CCK-8 assays showed that the miR-1246 did not influence cell growth (Fig. 1b) and transwell assays with or without Matrigel indicated that miR-1246 markedly induced migration and invasion in NSCLC cells (Additional file 2: Figure S2). Next, a miR-1246 expressing lentivirus vector was constructed to infect A549 and H226 cells which helps to establish stably transfected cell lines. In transwell assays, A549 cells overexpressing miR-1246 showed enhanced migratory and invasive abilities compared with vector control (Fig. 1c and d). Similar results were also observed in H226 cells (Fig. 1c and d). We further transfected A549 and H226 cells with miR-1246 inhibitors to confirm the findings above. The results showed that the miR-1246 inhibitor could significantly inhibit the migration and invasion of A549 and H226 cells (Fig. 1e and f). Taken together, these data demonstrated that miR-1246 can promote NSCLC cell migration and invasion.

**Fig. 1:** The miR-1246 is often upregulated in NSCLC and promotes NSCLC cell migration and invasion. **a** The relative expression of mature miR-1246 in 50 pairs of NSCLC tissues and their corresponding noncancerous lung tissues were measured using TaqMan real-time PCR and normalized to U6 snRNA. **b** CCK-8 assays of A549 and H226 cells were performed every other day after transfection with a miR-1246 mimic or negative control (nc). The data are presented as the mean ± S.E.M. **c**, **d** Transwell migration and invasion assays of A549 and H226 cells stably expressing miR-1246 or mock control. **e**, **f** Transwell migration and invasion assays for A549 and H226 cells transfected with either miR-1246 inhibitor or negative control. Representative images are shown on the left, and quantification is shown on the right. The results are representative of at least three independent experiments. * *p* < 0.05, ** *p* < 0.01, *** *p* < 0.001

RETRACTED

### The miR-1246 Can downregulate CPEB4 expression by directly targeting its 3’ UTR

To unravel the detailed molecular mechanisms for miR-1246 on NSCLC cell migration and invasion, mRNA microarray assays were performed to identify the genes that were suppressed by miR-1246 in both A549 and H226 cells transfected with the miR-1246 mimic. At the same time, potential targets were predicted using the algorithm TargetScan. By integrating the results of these two strategies, 17 genes were found to be plausible targets (Fig. 2a, Table 1). Real-time PCR, dual-luciferase reporter and western blot analysis were then performed to verify whether specific genes were actually targeted by miR-1246 (Fig. 2b-d). After preliminary screening, CPEB4 was confirmed as a potential target for miR-1246 (Fig. 2c and d).

**Fig. 2:** miR-1246 downregulates CPEB4 expression by directly targeting its 3’ UTR. **a** Scheme for the identification of candidate genes combining microarray assays and a target prediction algorithm. **b** The mRNA expression levels of the predicted genes in A549 and H226 cells expressing miR-1246 or vector were evaluated by real-time PCR. **c** Dual-luciferase activity assays were used to determine the binding potential between miR-1246 and the 3’ UTR of these candidate genes. Renilla luciferase activity was detected as an internal control. **d** Western blot assays of the TRAK2 and CPEB4 protein levels in A549, H226 and HEK 293 T cells. **e** The sequences of the putative miR-1246-binding site in the wild-type and mutant (underlined) *CPEB4* 3’ UTR. **f** The putative binding sequences for miR-1246 within the human (Has), chimpanzee (Ptr), rhesus (MMl) and mouse (Mmu) *CPEB4* 3’ UTR. Seed sequences are indicated as emphasized with shadow. **g** The relative luciferase activity of luciferase reporters with wild-type or mutant *CPEB4* 3’ UTRs was determined in HEK 293 T cells, which were co-transfected with the miR-1246 mimic or negative control (nc). Renilla luciferase activity was analyzed as an internal control. There is statistical significance between the wild-type group and the mutant group with miR-1246 transfection. **h** The protein levels of CPEB4 were determined by western blot assays in H226 cells infected with miR-1246 or mock vector and H226 cells transfected with the miR-1246 inhibitor or negative control (nc). * *p* < 0.05, ** *p* < 0.01, *** *p* < 0.001

**Table 1:** The possible target genes for miR-1246 in NSCLC cells

Gene	Official full name
*CPEB4*	Cytoplasmic polyadenylation element binding protein 4
*ARL2BP*	ADP-ribosylation factor-like 2 binding protein
*KLF12*	Kruppel-like factor 12
*RPS6KB1*	ribosomal protein S6 kinase, 70 kDa, polypeptide 1
*UGCGL1*	UDP-glucose glycoprotein glucosyltransferase 1
*RSBN1*	round spermatid basic protein 1
*HTR2A*	5-hydroxytryptamine (serotonin) receptor 2A
*TRAK2*	trafficking protein, kinesin binding 2
*GPR85*	protein-coupled receptor 85
*MRPL19*	mitochondrial ribosomal protein L19
*GALE*	UDP-galactose-4-epimerase
*PDAP1*	PDGFA associated protein 1
*ARSB*	Arylsulfatase B
*FAM55C*	family with sequence similarity 55, member C
*RBM24*	RNA binding motif protein 24
*CYLD*	cylindromatosis (turban tumor syndrome)
*PNPO*	pyridoxamine 5’-phosphate oxidase

The sequence analysis of the CPEB4 3’ UTR by TargetScan showed only one plausible site for miR-1246 binding. The site was also highly conserved among chimpanzees, rhesus, mice and humans (Fig. 2e and f). To further determine whether CPEB4 is directly regulated by miR-1246 via common 3’ UTR binding, a luciferase reporter containing the wild-type or mutant 3’ UTR of CPEB4 was constructed. After co-transfection with a miR-1246 mimic, the luciferase activities were significantly decreased in the group co-transfected with wild-type CPEB4 3’ UTR containing vector, while the luciferase activity was not reduced in the mutant 3’ UTR group (Fig. 2g). This result suggests that miR-1246 binds to the 3’ UTR of CPEB4 via the predicted binding site.

RETRACTED

In addition, immunoblots also showed that transfection with miR-1246 can result in decreased CPEB4 expression in H226 cells (Fig. 2h). Conversely, the miR-1246 inhibitor can increase the amount of CPEB4 (Fig. 2h). Collectively, these results indicated that miR-1246 could negatively modulate CPEB4 expression by directly targeting its 3’ UTR.

### CPEB4 is usually reduced in NSCLC

Previous reports indicated that CPEB4 plays a role in regulating translation, meiotic division and mitosis [22, 23]. However, the expression of CPEB4 in NSCLC remains unknown. The protein levels of CPEB4 were determined with IHC staining. The CPEB4 expression was relatively high in noncancerous adjacent tissues. In contrast, CPEB4 staining was relatively weak in NSCLC samples (Fig. 3a). Notably, the intrinsic CPEB4 expression exhibited close correlation with the overall survival of NSCLC patients (Fig. 3b). There was no correlation between CPEB4 levels and other clinicopathological factors such as age, sex and stage (Table 2). Taken together, these data suggested that the CPEB4 level was frequently downregulated in NSCLC, and its expression substantially affected NSCLC prognosis.

RETRACTED

**Fig. 3:** CPEB4 is often reduced in NSCLC and contributes to the low overall survival of NSCLC patients. **a** Immunohistochemical staining of CPEB4 in NSCLC tissues and noncancerous adjacent tissues. Two cases were shown. NAT: noncancerous adjacent tissue. **b** The survival curves are shown for low or high CPEB4 expression level (p < 0.01). The statistical analyses of cases in groups were performed with the *χ* ^2^ test and Kaplan-Meier plots. * *p* < 0.05, ** *p* < 0.01, *** *p* < 0.001

**Table 2:** Correlation between CPEB4 expression and different clinicopathological features in NSCLC^a^

Clinicopathological features	No. of cases	CPEB4 expression		*P*
		High (n, %)	Low (n, %)	
Age				
<60	26	13(50.0 %)	13(50.0 %)	0.496
≥60	24	11(45.8 %)	13(54.2 %)	
Gender				
Male	22	12(54.5 %)	10(45.5 %)	0.296
Female	28	2(42.9 %)	12(57.1 %)	
Histology/differentiation				
Well + Moderate	30	14(46.7 %)	16(53.3 %)	0.387
Poor	20	11(55.0 %)	9(45.0 %)	
TNM stage				
I + II	29	14(48.3 %)	15(51.7 %)	0.312
III + IV	21	12(57.1 %)	9(42.9 %)	

^a^The median level was used as the cutoff

### The miR-1246 functions via reducing CPEB4 level in NSCLC

To further clarify the effects of CPEB4 in NSCLC cells, siRNAs against *CPEB4* were intricately designed and transfected into 293 T cells. The knockdown efficiency of three constructs was first verified and the results showed that specific CPEB4 siRNAs could efficiently reduce *CPEB4* transcripts (Fig. 4a). The mRNA and protein levels of CPEB4 were markedly decreased, particularly in the si-CPEB4-1 group (Fig. 4a, b). Therefore, si-CPEB4-1 was used in further analysis. A549 cells were transfected with siRNAs and then subjected to transwell assays. The result showed that A549 cells transfected with *CPEB4* siRNA exhibited elevated migration and invasion (Fig. 4c). These results suggested that CPEB4 might be a direct target of miR-1246 in NSCLC.

**Fig. 4:** CPEB4 suppresses miR-1246-induced migration/invasion and its expression is inversely correlated with miR-1246 in NSCLC. **a**, **b** Real-time PCR and western blot of CPEB4 expression in HEK 293 T cells transfected with siRNAs targeting CPEB4 or a negative control (nc). **c** Transwell migration and invasion assays of A549 cells were performed after transfection with a miR-1246 inhibitor, CPEB4 siRNA or a negative control (nc). The protein level of CPEB4 was detected through western blot. There is statistical significance between group 1 and group 2 as well as between group 2 and group 4. The results are presented as the mean ± SD. **d** The relative expression of CPEB4 at the mRNA level was analyzed through real-time PCR (normalized to β-actin). **e** The correlation between *CPEB4* expression and mature miR-1246 in various lung cancer cell lines was analyzed by linear regression. **f** The mRNA level of *CPEB4* was determined in 50 pairs of NSCLC tissues and matched noncancerous adjacent lung tissues by real-time PCR. **g** The correlation between *CPEB4* expression and mature miR-1246 was analyzed in the same NSCLC samples by linear regression. The expression data were normalized to β-actin and U6 snRNA, respectively. * *p* < 0.05, ** *p* < 0.01, *** *p* < 0.001

We next attempted to determine whether CPEB4 was involved in miR-1246-induced NSCLC cell migration and invasion. The miR-1246 inhibitor and siRNAs targeting *CPEB4* were co-transfected into A549 cells. The subsequent transwell assays demonstrated that *CPEB4* knockdown partly neutralized the suppressive effects of the miR-1246 inhibitor on NSCLC cell migration and invasion (Fig. 4c). These data provided further evidence that CPEB4 could inhibit miR-1246-induced NSCLC cell migration and invasion, suggesting that CPEB4 is a direct and functional target of miR-1246 in NSCLC. We then evaluated the expression of *CPEB4* mRNA in various lung cancer cell lines (Fig. 4d). The results showed that the *CPEB4* mRNA was inversely correlated with the expression of miR-1246 in these cell lines (Fig. 4e and Additional file 1: Figure S1C). To extend our analysis to clinical cases, we assessed the mRNA level of *CPEB4* in the previous 50 cases of NSCLC and the adjacent noncancerous lung tissues. *CPEB4* mRNA was downregulated in NSCLC tissues compared with their respective noncancerous tissues (Fig. 4f), consistent with the observed CPEB4 protein levels. Moreover, the expression of *CPEB4* was inversely correlated with the level of miR-1246 in these NSCLC samples (Fig. 4g). These data suggested that *CPEB4* mRNA expression is negatively correlated with miR-1246 expression in NSCLC.

RETRACTED

## Discussion

MiRNAs are a class of small, noncoding RNAs which regulate gene expression by targeting mRNAs for translational repression or degradation. Accumulating evidence suggests that deregulation of miRNAs has been frequently observed in tumor tissues. These miRNAs have regulatory roles in the pathogenesis of cancer [24, 25]. Indeed, patients with lung cancer often exhibit tumor cell invasion and metastasis before diagnosis, which renders current treatments, including surgery, radiotherapy, and chemotherapy, ineffective. Therefore, studying the molecular basis of lung cancer is crucial for designing new therapeutic agents to improve the survival rate.

In current work, we found that the level of miR-1246 is frequently raised in NSCLC and promotes cell migration and invasion. CPEB4 serves as the direct miR-1246 target gene and is usually suppressed in NSCLC, and its expression is correlated with NSCLC patient outcome.

We found that the expression level of miR-1246 in NSCLC cells is relatively high (Fig. 1). To explore its functional role, we performed series of assays in NSCLC cell lines and found that inhibition of miR-1246 in A549 cells significantly reduce migration and invasion. However, simultaneous reduction in CPEB4 expression reverses the effect of miR-1246 inhibition suggesting that CPEB4 might be a functional target of miR-1246 in NSCLC. Recent reports also suggested that miR-1246 can enhance cell migration and invasion in hepatocellular carcinoma (HCC) cells [26] further extending the oncogenic role of miR-1246. Another recent report on miR-1246 demonstrated that miR-1246 is a novel target of p53 transcription factor and its analogue p63/p73 to suppress the expression of DYRK1A and activate NFAT both leading to possible tumorigenesis [27]. This finding further suggested a potential linkage of p53 family with Down syndrome. Therefore, current knowledge has unraveled an oncogenic role of miR-1246 in at least specific tumors. Further studies are strongly needed to unravel the hidden layer of complexity about miR-1246 and its implications in tumorigenesis.

The mechanistic insights into the biological role of miR-1246 on migration and invasion argued that the target gene CPEB4 might be implicated. CPEB4 belongs to the cytoplasmic polyadenylation element-binding protein family, the members of which primarily modulate translation by regulating the polyadenylation of target genes. The CPEB family commonly contains two subfamilies, CPEB1 and CPEB2. Although CPEB1 has been investigated in depth, the function of CPEB4 which is a member of the CPEB2 subfamily remains elusive. It was shown that CPEB4 servers as a pro-survival protein in neurons and contributes largely meiosis [28, 29]. In pancreatic ductal cancer and neuroblastoma, CPEB4 is upregulated leading to the growth and invasion of cancer cells [30]. In current study, we observed that the levels of CPEB4 were commonly down-regulated in NSCLC. The tissue-specific feature and some other unexplored factors might contribute to this phenomenon in distinct tumor tissues. Furthermore, we found that knockdown of *CPEB4* could promote the migration and invasion of NSCLC cells. This contradiction might be ascribed to the distinct downstream targets modulated by CPEB4 in different cells because CPEB4 can alter the translation of numerous genes by directly binding to the 3’ UTR [29]. Intriguingly, relatively high CPEB4 level exhibited a better survival in NSCLC patients. These results suggested that CPEB4 might act as a prognostic factor in NSCLC. We also demonstrated that miR-1246 and CPEB4 expression were inversely correlated in NSCLC samples suggesting that the downregulation of CPEB4 may be at least partially due to the upregulation of miR-1246. Targeting CPEB4 by microRNAs has also been reported previously [29]. The members of the CPEB2 subfamily can be controlled by microRNAs through a conserved sequence in their 3’ UTR [29]. Taken together, our findings demonstrate that regulation by microRNA may be a common strategy utilized in CPEB4 regulation. How CPEB4 is involved in the progression of lung cancer especially the molecular mechanisms demand in-depth investigation.

RETRACTED

## Conclusions

In summary, our findings demonstrated that elevated miR-1246 expression may increase the migratory and invasive potential of NSCLC cells. Knockdown of the miR-1246 target gene *CPEB4* enhanced the migration and invasion of NSCLC cells. Importantly, CPEB4 expression is correlated with NSCLC patient outcome. Therefore, miR-1246/CPEB4 may denote a promising prognostic and therapeutic target in NSCLC.

## Additional files

Additional file 1: Figure S1. Transfection efficiency and endogenous expression of miR-1246. (A) The relative expression level of mature miR-1246 was determined in A549 and H226 cells infected with pWPXL-miR-1246 or control lentivirus. U6 snRNA was used as an internal control. (B) The relative expression of miR-1246 was determined in A549 and H226 cells infected with miR-1246 inhibitor or control. (C) The relative expression of miR-1246 in various lung cancer cells. The relative expression level of mature miR-1246 was detected by TaqMan real-time PCR. The data were normalized to U6 snRNA. (TIFF 262 kb) Additional file 2: Figure S2. A miR-1246 mimic facilitates NSCLC cell migration and invasion in vitro. (A) Transwell migration assays of A549 and H226 cells transfected with the miR-1246 mimic or negative control (NC). (B) Transwell invasion assays of A549 and H226 cells transfected with the miR-1246 mimic or NC. The values shown indicate the mean ± S.E.M. * *p* < 0.05, ** *p* < 0.01, *** *p* < 0.001. (TIFF 1195 kb)

## References

[1] Jemal A, Siegel R, Xu J, Ward E (2010). Cancer statistics, 2010. CA Cancer J Clin.

[2] Lewis BP, Burge CB, Bartel DP (2005). Conserved seed pairing, often flanked by adenosines, indicates that thousands of human genes are microRNA targets. Cell.

[3] Fabbri M (2010). miRNAs as molecular biomarkers of cancer. Expert Rev Mol Diagn.

RETRACTED

[4] Baranwal S, Alahari SK (2010). miRNA control of tumor cell invasion and metastasis. Int J Cancer.

[5] Fortunato O, Boeri M, Verri C, Moro M, Sozzi G (2014). Therapeutic use of MicroRNAs in lung cancer. Biomed Res Int.

[6] Weidhaas JB, Babar I, Nallur SM, Trang P, Roush S, Boehm M, Gillespie E, Slack FJ (2007). MicroRNAs as potential agents to alter resistance to cytotoxic anticancer therapy. Cancer Res.

[7] Wang R, Wang ZX, Yang JS, Pan X, De W, Chen LB (2011). MicroRNA-451 functions as a tumor suppressor in human non-small cell lung cancer by targeting ras-related protein 14 (RAB14). Oncogene.

[8] Qi L, Bart J, Tan LP, Platteel I, Sluis T, Huitema S, Harms G, Fu L, Hollema H, Berg A (2009). Expression of miR-21 and its targets (PTEN, PDCD4, TM1) in flat epithelial atypia of the breast in relation to ductal carcinoma in situ and invasive carcinoma. BMC Cancer.

[9] Adams BD, Kasinski AL, Slack FJ (2014). Aberrant regulation and function of microRNAs in cancer. Curr Biol.

[10] Ishiguro H, Kimura M, Takeyama H (2014). Role of microRNAs in gastric cancer. World J Gastroenterol.

[11] Calin GA, Sevignani C, Dumitru CD, Hyslop T, Noch E, Yendamuri S, Shimizu M, Rattan S, Bullrich F, Negrini M, Croce CM (2004). Human microRNA genes are frequently located at fragile sites and genomic regions involved in cancers. Proc Natl Acad Sci U S A.

[12] Calin GA, Dumitru CD, Shimizu M, Bichi R, Zupo S, Noch E, Aldler H, Rattan S, Keating M, Rai K (2002). Frequent deletions and down-regulation of micro- RNA genes miR15 and miR16 at 13q14 in chronic lymphocytic leukemia. Proc Natl Acad Sci U S A.

[13] Michael MZ, O’ Connor SM, van Holst Pellekaan NG, Young GP, James RJ (2003). Reduced accumulation of specific microRNAs in colorectal neoplasia. Mol Cancer Res.

[14] Takamizawa J, Konishi H, Yanagisawa K, Tomida S, Osada H, Endoh H, Harano T, Yatabe Y, Nagino M, Nimura Y (2004). Reduced expression of the let-7 microRNAs in human lung cancers in association with shortened postoperative survival. Cancer Res.

[15] Metzler M, Wilda M, Busch K, Viehmann S, Borkhardt A (2004). High expression of precursor microRNA-155/BIC RNA in children with Burkitt lymphoma. Genes Chromosomes Cancer.

[16] Lim EL, Trinh DL, Scott DW, Chu A, Krzywinski M, Zhao Y, Robertson AG, Mungall AJ, Schein J, Boyle M (2015). Comprehensive miRNA sequence analysis reveals survival differences in diffuse large B-cell lymphoma patients. Genome Biol.

[17] Hayashita Y, Osada H, Tatematsu Y, Yamada H, Yanagisawa K, Tomida S, Yatabe Y, Kawahara K, Sekido Y, Takahashi T (2005). A polycistronic microRNA cluster, miR-17-92, is overexpressed in human lung cancers and enhances cell proliferation. Cancer Res.

RETRACTED

[18] Borkowski R, Du L, Zhao Z, McMillan E, Kosti A, Yang CR, Suraokar M, Wistuba II, Gazdar AF, Minna JD (2015). Genetic mutation of p53 and suppression of the miR-17 approximately 92 cluster are synthetic lethal in non-small cell lung cancer due to upregulation of vitamin D Signaling. Cancer Res.

[19] Zhang Y, Liao JM, Zeng SX, Lu H (2011). p53 downregulates Down syndrome-associated DYRK1A through miR-1246. EMBO Rep.

[20] Zhang Y, Liu D, Chen X, Li J, Li L, Bian Z, Sun F, Lu J, Yin Y, Cai X (2010). Secreted monocytic miR-150 enhances targeted endothelial cell migration. Mol Cell.

[21] Zhang S, Shan C, Kong G, Du Y, Ye L, Zhang X (2012). MicroRNA-520e suppresses growth of hepatoma cells by targeting the NF-kappaB-inducing kinase (NIK). Oncogene.

[22] Huang YS, Kan MC, Lin CL, Richter JD (2006). CPEB3 and CPEB4 in neurons: analysis of RNA-binding specificity and translational control of AMPA receptor GluR2 mRNA. EMBO J.

[23] Igea A, Mendez R (2010). Meiosis requires a translational positive loop where CPEB1 ensues its replacement by CPEB4. EMBO J.

[24] Dykxhoorn DM (2010). MicroRNAs and metastasis: little RNAs go a long way. Cancer Res.

[25] Hummel R, Hussey DJ, Haier J (2010). MicroRNAs: predictors and modifiers of chemo- and radiotherapy in different tumour types. Eur J Cancer.

[26] Sun Z, Meng C, Wang S, Zhou N, Guan M, Bai C, Lu S, Han Q, Zhao RC (2014). MicroRNA-1246 enhances migration and invasion through CADM1 in hepatocellular carcinoma. BMC Cancer.

[27] Liao JM, Zhou X, Zhang Y, Lu H (2012). MiR-1246: a new link of the p53 family with cancer and Down syndrome. Cell Cycle.

[28] Kan MC, Oruganty-Das A, Cooper-Morgan A, Jin G, Swanger SA, Bassell GJ, Florman H, van Leyen K, Richter JD (2010). CPEB4 is a cell survival protein retained in the nucleus upon ischemia or endoplasmic reticulum calcium depletion. Mol Cell Biol.

[29] Morgan M, Iaconcig A, Muro AF (2010). CPEB2, CPEB3 and CPEB4 are coordinately regulated by miRNAs recognizing conserved binding sites in paralog positions of their 3’-UTRs. Nucleic Acids Res.

[30] Ortiz-Zapater E, Pineda D, Martinez-Bosch N, Fernandez-Miranda G, Iglesias M, Alameda F, Moreno M, Eliscovich C, Eyras E, Real FX (2012). Key contribution of CPEB4-mediated translational control to cancer progression. Nat Med.

